The article "Prediction Model Construction for Ischemic Stroke Recurrence with BP Network and Multivariate Logistic Regression and Effect of Individualized Health Education" was published in 2022. Journal: Comput Math Methods Med.

# Prediction Model Construction for Ischemic Stroke Recurrence with BP Network and Multivariate Logistic Regression and Effect of Individualized Health Education

**DOI:** 10.1155/2022/4284566

**Published:** 2022-06-22

**Authors:** Ting Lu, Yun Wang

**Affiliations:** Department of Neurology Nursing, Sichuan Provincial People's Hospital, University of Electronic Science and Technology of China, Chinese Academy of Sciences Sichuan Translational Medicine Research Hospital, Chengdu, Sichuan 610072, China

## Abstract

Stroke is an acute cerebrovascular disease caused by the rapid rupture or blockage of intracranial blood vessels for a variety of reasons, preventing blood from flowing into the brain and causing damage to brain tissue. The global burden of stroke disease is quickly increasing, and ischemic stroke (IS) accounts for 60 percent to 70 percent of all strokes, owing to the prevalence of people's bad lifestyles and the intensity of global ageing. Although most IS patients have received effective treatment, many patients still have certain dysfunction or death after treatment, and the recurrence rate is about 18%, which brings a heavy economic burden to society and families. Therefore, it is urgent to build a postoperative prediction model for IS, so as to take targeted clinical intervention measures, which has extremely important practical significance for improving the prognosis of IS. The following work has been done in this paper: (1) the theoretical background for the BP prediction model and logistic regression prediction model suggested in this work is offered, as well as the research progress and related technologies of IS recurrence prediction by domestic and foreign academics. (2) The basic principles of BPNN and logistic regression are introduced, and the logistic multifactor predictor is constructed. (3) The experimental results show that the consistency rate, sensitivity, and specificity of the prediction results of BPNN are higher than those of logistic regression, indicating that for diseases such as IS, which have many pathogenic factors and complex relationships between factors, the fitting effect of BPNN model is better than that of the logistic regression model.

## 1. Introduction

Stroke follows cardiovascular disease as the major cause of mortality globally. There are about 2.4 million new stroke patients in my country every year, about 1.1 million deaths, and about 11 million poststroke survivors, of which about 70% are IS. IS refers to the ischemic necrosis or softening of the brain tissue caused by ischemia and hypoxia caused by various reasons. About 75% of IS patients have different degrees of dysfunction after the onset of the disease, which brings a heavy burden to the family and society, and IS is prone to relapse within 1 year after the onset of IS. The recurrence rates were 10.9%, 13.4%, and 14.7%, respectively [1]. In the first year after the onset of acute ischemic stroke, 1 in 18 people has a recurrent stroke. The harm caused by the recurrence of IS is far greater than that of the first stroke. The neurological damage caused by the recurrent stroke is more serious and more refractory and has a higher mortality rate than the first stroke. It is one of the main causes of death, rehospitalization, and long-term disability. Cumulative mortality after relapse more than doubled compared with first-episode stroke, and the risk of death increased approximately 17-fold. Reducing the recurrence rate of IS is the key to improving the prognosis of stroke, and secondary prevention of stroke can reduce the risk of IS recurrence by about 13% to 67%. Risk prediction of IS recurrence is the key to effective clinical secondary prevention and the most effective means to reduce the fatality and disability rate of patients [2, 3]. There are two main issues to consider in IS recurrence risk prediction: the first is the selection of IS recurrence risk predictors. The screening of predictive factors is an important step in the construction of predictive models, and the effect of predictive models depends on the accuracy and sensitivity of the predictive factors. There are many studies on the risk factors of IS recurrence, but the research results are affected by regions, medical policies, social economy, etc., and the research results are different.

It is difficult to predict the screening of IS recurrence risk factors. The risk prediction of IS recurrence is mainly based on clinical factors. The results of risk verification showed that the AUC values of the area under the ROC curve were all 0.59. The model did not cover all risk factors and had a limited predictive impact, making it difficult to meet clinical needs [4]. Scholars have increasingly employed biomarkers, imaging markers, and TCM syndrome distinguishing signals to the risk prediction of IS recurrence, improving the prediction effect in recent years. The method for building the IS recurrence risk prediction model is the second. Traditional statistical methods for developing prediction models, such as Cox proportional hazards regression analysis and logistic regression analysis, are currently the most popular. Traditional statistical methods, on the other hand, have stringent data-type restrictions and have little impact on data mining when dealing with clinical recurrence data. Machine learning has started to be used to illness risk prediction with the progress of computer technology and smart medical care. Multidisciplinary in nature, machine learning draws on a variety of fields, including probability and statistics, approximation theory, convex analysis, and theory of algorithm complexity. The artificial intelligence of a computer may be realized via the machine's ability to learn from the data's inherent regularity information and gain new experience and knowledge [5, 6]. Machine learning algorithms have the characteristics of high efficiency and accuracy in processing big data, and the prediction effect is better than traditional statistical methods [7]. The disease risk prediction model built with BPNN, SVM algorithm, XGBoost algorithm, and other machine learning algorithms outperforms established statistical methods such as the logistic regression model and the Cox proportional hazards regression model [8]. As a result, this work used prospectively gathered medical-related data from IS patients, applied multivariate analysis to screen out risk factors affecting IS prognosis, and built a machine learning algorithm-based risk prediction for ischemic stroke with a bad prognosis. The model can quickly predict and identify the risk of poor functional recovery of IS patients in the early stage of disease diagnosis and treatment, scientifically assist the selection of clinical treatment plans, improve the prognosis of stroke patients, reduce the disability rate of stroke, and improve the quality of medical care, and it provides a new idea for predicting the prognosis of IS.

The following is the paper's organisation paragraph: in Section 2, the related work is provided. The suggested work's approaches are examined in Section 3. The experiments and results are discussed in Section 4. Finally, the research is completed in Section 5.

## 2. Related Work

A large number of studies have shown that the prognosis of ischemic stroke is affected by factors such as age, family history, smoking, drinking, hypertension, abnormal lipid metabolism, abnormal glucose metabolism, and hyperhomocysteinemia. This provides a good basis for the risk prediction study of poor prognosis of ischemic stroke [9, 10]. At present, traditional evaluation tools, such as Essen scale, ABCD2 scale, and SPI-II scale, are mainly used in clinical practice for ischemic stroke to predict the recurrence risk of patients. ESRS is based on the stroke prediction model developed by the CAPRIE Institute. The higher the score, the greater the risk of stroke recurrence. The Essen score is currently the most commonly used scale in the world to predict the long-term recurrence risk of stroke [11]. Reference [12] developed the ABCD2 scoring method based on the ABCD scoring system proposed by the “Oxfordshire Community Stroke Project” study to assess the risk of stroke in patients with transient ischemic attack. Reference [13] proposed the SPI-III scale in 2000 to assess the long-term recurrence risk of stroke patients. Age over 70, diabetes, coronary heart disease, and a history of stroke are all listed as risk factors for stroke recurrence in the evaluation tool. Using manual or traditional statistical analysis methods, the above-mentioned scoring scales combine several risk factors that affect stroke prognosis and assign varying weights to each risk factor. Diverse groups of people have different lifestyles; thus, it is still unclear whether the weights allocated to these aspects are appropriate for Chinese people. At present, for the prediction of IS prognosis, domestic and foreign scholars still mostly use retrospective cohort studies to construct a risk prediction model for poor stroke prognosis based on traditional statistical analysis of logistic regression and Cox regression [14, 15]. The medical and health sector has entered the age of big data as a result of the fast growth of medical and health informatization building. Machine learning algorithms have been extensively employed in the medical industry, such as illness prediction, disease prognosis evaluation, disease auxiliary diagnosis, and health management, in the face of these large data with huge volume, varied kinds, and high hidden value [16]. This is because machine learning algorithms can take into account more variables and effectively reflect the unpredictable and complex nature of the human body than traditional prediction models that only consider one or two variables. A multilayer feedforward neural network known as the BPNN was initially suggested by researchers in 1986, and it has since become the most widely used neural system model in neuroscience [17]. BPNN does not have high requirements for data types and has strong nonlinear mapping ability and adaptive ability, which can effectively dig out the influencing factors related to the occurrence of diseases from the complicated medical big data and scientifically evaluate the occurrence of disease risk [18]. Reference [19] used BPNN and logistic regression model to construct a risk prediction model for spontaneous hemorrhagic transformation in ischemic stroke patients, respectively. The results showed that the predictive performance of BPNN was better than that of the logistic regression model. Random forest is a supervised learning ensemble algorithm proposed by reference [19] in 1995. Because of its great antinoise capabilities and difficult overfitting, the algorithm is commonly employed in illness risk prediction. The random forest model outperforms the BPNN model and the logistic regression model in predicting the risk of coronary stenosis, according to academic research, and its AUC values are 0.752, 0.723, and 0.739, respectively. Based on the current research status at home and abroad, various traditional risk scale scores have achieved certain results in the prognosis prediction of ischemic stroke, but various scales only include simple indicators such as age and past medical history, and the prediction accuracy is often low and cannot fully explain whether there is an interaction between the indicators. In addition, the existing studies also have problems such as small sample size, single center, retrospective studies, and low data quality and sample representativeness [20]. Because of the fast growth of data mining technology and the increasing amount of data in electronic medical records, the use of machine learning in the area of illness prognostic prediction has made significant strides [21–24]. There are still few studies on prognosis prediction of hemorrhagic stroke patients, and further research is needed.

## 3. Method

### 3.1. The Basic Principle of Artificial Neural Network

Analogous neural networks (ANNs) are mathematical models of the brain's synaptic connections. Modern neuroscience research has resulted in the reduction, abstraction, and modeling of the structure and function of the biological nerve system of the human brain, which reflects the human brain's essential properties. This nonlinear network system is made up of a large number of small basic units called neurons that are connected in a way that resembles how the human brain processes information and distributes processing. ANN does not use mathematical methods for precise calculation, nor does it need to predetermine basic functions like regression equations, but directly train the neural network with data or signal samples, and obtain a response after a limited number of iterative calculations. Another advantage of the neural network method is that it requires no prior information and offers self-learning, self-adaptation, and fault tolerance, making it ideal for multivariate pattern identification. It provides a new way to solve the uncertainty, ambiguity, and dynamic complexity in hygiene evaluation. At present, it has been widely used in the prediction, diagnosis, image processing, and other aspects of diseases in the medical field, especially the error backpropagation algorithm which is more widely used.

#### 3.1.1. Backpropagation BP Network Algorithm

The error backpropagation technique was first published by Paul Werbos in 1974, although it was not extensively used at the time. BPNN is a multilayer forward neural network based on this approach. It was not until the mid-1980s that some scholars conducted further research on the BP algorithm and wrote the BP algorithm into the book “Parallel Distributed Processing,” and the BP algorithm was not widely known. BPNN is a typical multilayer feedforward neural network using a teacher-supervised learning algorithm. It has powerful computing power and can master the input-output mapping relationship implied by the learning sample through training and has a wide range of applications in classification and prediction. Parallel networks are used in the BPNN. Hidden node output signals are passed to the output node, and eventually, the output result is supplied. Forward propagation and backward propagation of errors are both used in the algorithm's learning phase. A forward propagation method is used to process input information from the input layer to the hidden layer and transmit it to the output layer. A neuron's current state solely influences the following neuron's current state. In the event that the desired output result cannot be attained in the output layer, the error signal is returned over the original connection channel and is then processed via backpropagation. The mean square of the error is reduced by adjusting the weights of neurons in each layer. BPNN's excellent nonlinear mapping ability and generalization function have been shown by neural network theory. A three-layer network may realize any continuous function or mapping.

#### 3.1.2. BP Network Structure

BPNN is by far the most famous and widely used neural network. Theoretically, the complex nonlinear relationship can be fully described by a three-layer feedforward network. An input layer, a hidden layer, and an output layer are the three layers that make up a network. The topology of a typical BPNN is shown in Figure 1.

Because of this, the BP algorithm alters its weights and biases in the opposite direction of gradient, which is similar to how a linear network's learning algorithm works. A mathematical formula for the BP algorithm's iterative computation is as follows:

(1) $$\begin{array}{c} x_{k+1}=x_{k}-\nu g_{r}, \end{array}$$

where *x*_*k*_ represents the current weight and bias, *x*_*k*+1_ represents the next weight and bias generated by iteration, *g*_*r*_ is the gradient of the current error function, and *ν* represents the learning rate.

Using an example of a BPNN with two hidden layers and four total layers of neurons, we can figure out how the learning process works in this section. *M* is the number of inputs, and *m* is the identifier for any one of them. An *I* represents one of the *I* neurons in the first hidden layer, which has *I* neurons in total. There are a total of *j* neurons in the second hidden layer, each of which has been labeled with *j*. There are *P* neurons in the output layer, each of which is symbolized by the letter *p*. *w*_*mi*_ is the weight between the *m*th neuron in the input layer and the first hidden layer, which is indicated as the weight output from the *m*th neuron to the first hidden layer. *w*_*ij*_ Denotes the weight between the first and second hidden layers. Input and output weights are indicated by *w*_*ip*_ and *w*_*jp*_, respectively.

The neuron input is denoted as *Z*, the output is denoted as *O*, and *Z*_*i*_^*I*^ represents the input of the *i*^th^ neuron in the first hidden layer. Let the transfer function of all neurons be the sigmoid function. The training sample set is *X* = (*X*_1_, *X*_2_ ⋯ *X*_*N*_), and any training sample *X*_*k*_ is an *M*-dimensional vector, that is, *X* = (*X*_*k*1_, *X*_*k*2_ ⋯ *X*_*km*_)(k = 1, 2, ⋯, N); the expected response is *d*_*k*_, and the actual output is *Y*_*k*_. Let *n* be the number of iterations, and both the weights and the actual output are functions of *n*. When the network input training sample is *X* = (*X*_*k*1_, *X*_*k*2_ ⋯ *X*_*km*_), the network signal is transmitted in a forward manner. For the intermediate value of each layer, the expression can be written as follows.

The input of the *i*^th^ neuron in the first hidden layer is

(2) $$\begin{array}{c} Z_{i}^{I}=\overset{M}{\underset{m=1}{\sum }}w_{mi}x_{km}. \end{array}$$

The output of the *i*^th^ neuron in the first hidden layer is

(3) $$\begin{array}{c} O_{i}^{I}=f\left(\overset{M}{\underset{m=1}{\sum }}w_{mi}x_{km}\right). \end{array}$$

The output of the *j*^th^ neuron in the second hidden layer is

(4) $$\begin{array}{c} O_{i}^{I}=f\left(\overset{I}{\underset{i=1}{\sum }}w_{ij}O_{i}^{I}\right). \end{array}$$

The input of the *p*^th^ neuron in the output layer is

(5) $$\begin{array}{c} Z_{p}^{P}=\overset{J}{\underset{j=1}{\sum }}w_{jp}O_{j}^{J}. \end{array}$$

The output of the *p*^th^ neuron in the output layer, that is, the network output, is

(6) $$\begin{array}{c} y_{kp}=O_{p}^{P}=f\left(\overset{J}{\underset{j=1}{\sum }}w_{jp}O_{j}^{J}\right). \end{array}$$

The output error of the *p*^th^ neuron in the output layer is

(7) $$\begin{array}{c} e\left(n\right)=d_{kp}\left(n\right)-y_{kp}\left(n\right). \end{array}$$

Define the error energy as *e*, and the sum of the error energy of all neurons in the output layer is

(8) $$\begin{array}{c} E\left(n\right)=\frac{1}{2}\overset{P}{\underset{p=1}{\sum }}e^{2}\left(n\right). \end{array}$$

The error is opposite to the signal and propagates from back to front, and in the process of backpropagation, the weights and biases are modified layer by layer. The adjustment process of backpropagation and error is calculated below.

#### 3.1.3. Weight Adjustment

A partial differential of output error energy compared to the predicted response to weight is used in the BP algorithm, and the sign of this difference is used to alter weight. Following is the calculation of this partial differential's value. According to the learning rule of gradient descent, the correction amount of *w*_*jp*_ is

(9) $$\begin{array}{c} \Delta w_{jp}\left(n\right)=-\lambda \frac{\partial E\left(n\right)}{\partial w_{jp}\left(n\right)}=\theta_{p}^{P}\left(n\right)∙O_{j}^{J}\left(n\right), \end{array}$$

where *λ* is the learning step size, *p* is the local gradient, and *θ*_*p*_^*P*^(*n*) can be obtained according to the forward propagation process of the signal. Thus, the next iteration value of *w*_*jp*_ is calculated.

Get the next iteration value of the weight *w*_*jp*_(*n* + 1) before the hidden layer *J* and the output layer *P*:

(10) $$\begin{array}{c} w_{jp}\left(n+1\right)=w_{jp}\left(n\right)+∆w_{jp}\left(n\right). \end{array}$$

In the same way, the next iteration value of the weight *w*_*jp*_(*n*) before the hidden layer *I* and the hidden layer *J* can be obtained:

(11) $$\begin{array}{c} w_{ij}\left(n+1\right)=w_{ij}\left(n\right)+∆w_{ij}\left(n\right). \end{array}$$

Through the following iterative formula, the weight between the input layer *M* and the hidden layer *I* of the next iteration can be obtained.

(12) $$\begin{array}{c} w_{mi}\left(n+1\right)=w_{mi}\left(n\right)+∆w_{mi}\left(n\right). \end{array}$$

The above is the weight iteration formula of the learning rule of the full sigmoid transfer function BPNN including two hidden layers.

### 3.2. Basic Principles of Logistic Regression

#### 3.2.1. Logistic Regression Model

One way to look at the connection between binary data and some of their influencing elements is through a probabilistic nonlinear regression approach known as logistic regression (LR). It is often used in epidemiological research to examine the quantitative association between illnesses and other risk variables. Let the dependent variable *Y* be a binary variable whose value is

(13) $$\begin{array}{c} Y=\left\{\begin{array}{c} \;1,\;\text{negative result},\\ 0,\;\text{positive result}. \end{array}\right. \end{array}$$

There are also *m* independent variables (*X*_1_, *X*_2_ ⋯ *X*_*m*_) that affect the value of *Y*. Note that *P* = *P*(*Y* = 1|*X*_1_, *X*_2_ ⋯ *X*_*N*_) represents the probability of a positive result under the action of *m* independent variables, and the logistic regression model can be expressed as

(14) $$\begin{array}{c} P=\frac{1}{1+\exp\left(\alpha_{0}+\alpha_{1}X_{1}+\alpha_{2}X_{2}+\cdots +\alpha_{m}X_{m}\right)}, \end{array}$$

where *α*_0_ is the constant term and *α*_1_, *α*_2_, ⋯, *α*_*m*_ is the regression coefficient. If *L* is used to represent the linear combination of *m* independent variables,

(15) $$\begin{array}{c} L=\alpha_{0}+\alpha_{1}X_{1}+\alpha_{2}X_{2}+\cdots +\alpha_{m}X_{m}. \end{array}$$

Transforming formula (14), the logistic regression model can be expressed as the following linear form:

(16) $$\begin{array}{c} \ln\left(\frac{P}{1-P}\right)=\alpha_{0}+\alpha_{1}X_{1}+\alpha_{2}X_{2}+\cdots +\alpha_{m}X_{m}. \end{array}$$

The left end of formula (16) is the natural logarithm of the ratio of the probability of positive and negative results, which is called the logit transformation of *P*, and is recorded as logit*P*. It can be seen that although the value range of probability *P* is between 0 and 1, logit*P* has no numerical limit.

#### 3.2.2. Logistic Regression Modeling

A logistic regression model was developed using 500 patients acquired from a retrospective investigation as training samples. To examine the prediction performance, 200 patients from a prospective inquiry were employed as prediction samples, which were substituted into the developed model. Using the selected training samples, univariate logistic regression analysis was performed on the patients' basic information, clinical information, clinical biochemical indicators, postdischarge rehabilitation, and living conditions. For factor logistic regression model, see Table 1. Multifactor screening was carried out, and the forward method based on partial maximum likelihood estimation was used. With *α* = 0.05 as the inclusion criterion and *α* = 0.10 as the exclusion criterion, a logistic regression model for predicting the recurrence of ischemic stroke patients was established. There are 7 factors that finally entered the model (see Table 2).

## 4. Experiment and Analysis

### 4.1. Multivariate Logistic Regression Results

From the 7 influencing factors screened above, a logistic regression model is established, and its expression is logit(*P*) = −6.765 + 0.045*x*_1_ + 0.047*x*_2_ + 0.762*x*_3_ + 0.488*x*_4_ − 0.216*x*_5_ − 0.181*x*_6_ − 0.344*x*_7_; in the formula,*x*_1_,*x*_2_,*x*_3_,*x*_4_,*x*_5_,*x*_6_, and*x*_7_represent 7 factors of age, diastolic blood pressure, language barrier, alcohol consumption, triglyceride, aspirin, and sleep, respectively. Substitute 200 test samples into the logistic model established above, draw the ROC curve as shown in Figure 2, and calculate the area under the curve (AUC): AUC is 0.735, the prediction accuracy rate is 82.5%, and the sensitivity and specificity are 63.2% and 75.6%, respectively. Youden index is 38.2% (see Table 3).

### 4.2. BP Neural Network Modeling Results

#### 4.2.1. Establishment and Training of the Network Model

500 retrospectively investigated cases were used as the training set, and 200 prospectively investigated patients were used as the testing set. In order to simplify the calculation and prevent unnecessary overfitting, logistic regression was used to screen all factors by single factor in this study, and all 16 factors screened out by a single factor were used as input variables, that is, the input layer neurons *n* = 16. Modeling is done using three distinct types of simple BPNN models with varied amounts of hidden layers. The number of hidden layer nodes is calculated using the trial and error method in this study, with the first hidden layer node being defined as 8 and the second and third layers being reduced layer by layer to 6 and 3, respectively. At the same time, the maximum training error is to be selected as 0.001, the initial learning rate is 0.15, the minimum learning rate is 0.001, the maximum learning rate is 0.2, and the kinetic energy term *α* = 0.95.

#### 4.2.2. BP Neural Network Modeling Results

There is no statistically significant difference between the prediction results of the training set and the actual results of each model (*P* > 0.05), and the kappa values are all greater than 0.7, indicating that the prediction results are more consistent with the actual results. See Figure 3, so it can also be considered that the number of different hidden layers has little effect on the prediction results of the test set samples.

#### 4.2.3. Comparison of the Area under the ROC Curve of the Three BPNN Models

The predicted probability and actual results of the three BPNN models are used to make the ROC curve. The experimental results are shown in Figure 4. It can be seen that the prediction accuracy of BPNN-1 is higher than that of the other two models.

#### 4.2.4. Comparison of Prediction Accuracy and Validity of Models with Different Numbers of Hidden Layers

The prediction accuracy rates of each model are 95.2%, 94.5%, and 93.7%, respectively, and there is no statistical significance between the three accuracy rates. It can be seen that there is no difference in the prediction accuracy of the BPNN with different hidden layers. The results are shown in Figure 5.

#### 4.2.5. Analysis of Influencing Factors of BPNN

Increasing the number of hidden layers cannot improve the prediction effect of BPNN and may even affect the accuracy of model prediction. At the same time, the modeling time of a single hidden layer is short, and overfitting is not easy to occur. Choose a BPNN with one hidden layer. According to the influence degree of the imported influencing factors on the network, the top three influencing factors with the highest degree of influence are ADL, diastolic blood pressure, and aspirin consumption.

#### 4.2.6. Predictive Validity and Area under the ROC Curve of the Test Set of the BPNN Model

Substitute the data of the test set into the trained neural network model, and draw the ROC curve. The area under the ROC curve was calculated to be 0.796, and the calculated agreement of the model prediction was 86.8%, the sensitivity was 82.1%, the specificity was 80.5%, and the Youden index was 64.7%. The specific results are shown in Table 4.

### 4.3. Comparison Results between BP Neural Network and Logistic Regression

Compared with the logistic regression prediction model, the product under the ROC curve of the BPNN prediction result was 0.796, which was greater than the 0.735 obtained by the logistic regression prediction model, and the difference was statistically significant when comparing the area under the curve of the two models. The accuracy rate, sensitivity, specificity, and Youden index of the BPNN are also higher than those of the logistic regression model, so the prediction effect of the BPNN is better than that of the logistic regression, as shown in Figure 6.

## 5. Conclusion

The continuous development of my country's social economy has improved the living standards of residents. Because of the prevalence of unhealthy lifestyles in my country, the incidence of stroke has continued to climb, and the age of onset has gradually decreased. Stroke has had a significant impact on our people's health. In my country, it has become one of the most serious public health issues. The latest data from the Global Burden of Disease Study show that from 2005 to 2017, the incidence of ischemic stroke in my country was on the rise. In 2017, there were 156 new ischemic strokes per 100,000 people in my country. Research shows that the disability-adjusted life years lost due to stroke in my country ranks first among all diseases, with a recurrence rate of 9.7% within three months of onset and a disability rate of 37.1%. Because BPNN has been paid more and more attention by medical workers in disease prediction, people often use it to compare with the logistic regression model. The advantages of the logistic regression model are that it is simple and easy to use, the quantitative interpretation of the individual effects of factors is clear, the approximate estimation of the relative risk can be directly obtained, and the methodology of the quantitative dependence of variables can be established. The neural network model uses the information theory method, along with a human-like thinking mode, to develop the network by learning existing examples. It has a strong ability to solve the collinear effect and interaction between variables, and it has no restrictions on the distribution of data and can make full use of data information, with strong fault tolerance. As a nonlinear mathematical model, neural networks aid in the discovery of undiscovered correlations among various variables. Therefore, the following work is done in this paper: (1) the research progress and related technologies of IS recurrence prediction by domestic and foreign scholars are introduced, and the theoretical basis for the BP prediction model and logistic regression prediction model proposed in this paper is provided. (2) The basic principles of BPNN and logistic regression are introduced, and the logistic multifactor predictor is constructed. (3) The experimental results are that the area under the ROC curve of the logistic regression prediction model is 0.735, and the area under the ROC curve of the BPNN prediction results is 0.796. The Youden indices of BPNN and logistic regression are 64.7% and 38.2%, respectively, indicating that the prediction effect of BPNN is better than that of logistic regression. The consistency rate, sensitivity, and specificity of BPNN prediction results are greater than those of logistic regression, showing that the BPNN model has a superior fitting effect for disorders like ischemic stroke, which have many pathogenic components and complex connections between them.

## Figures and Tables

**Figure 1:** BP algorithm network structure.

**Figure 2:** ROC curve of test set multivariate logistic regression.

**Figure 3:** Result comparison of BP models with different numbers of hidden layers.

**Figure 4:** AUC and standard errors of BP models with different hidden layers.

**Figure 5:** Prediction accuracy indicator of BP models with different hidden layers.

**Figure 6:** Comparison of various indicators between the BP model and logistic regression.

**Table 1:** 16-item univariate logistic regression results.

Factors	*B*	S.E.	Wald	*P*	OR	OR (95% CI)
Age	0.045	0.006	23.12	<0.001	1.036	1.018-1.055
Systolic pressure	0.025	0.003	20.65	<0.001	1.015	1.005-1.028
Diastolic pressure	0.047	0.005	35.78	<0.001	1.040	1.022-1.055
Language disability	0.762	0.180	12.54	<0.001	2.169	1.460-2.221
CA	0.518	0.170	6.57	0.006	1.698	1.142-2.515
Hypertension	0.529	0.165	7.02	0.005	1.712	1.162-2.522
Hyperlipidemia	0.785	0.327	4.28	0.010	2.216	1.120-4.375
Smoking	0.219	0.096	4.18	0.011	1.289	1.028-1.627
Drinking	0.488	0.205	4.30	0.010	1.661	1.073-2.572
ADL	0.327	0.104	8.53	0.002	1.428	1.131-1.815
Triglycerides	0.216	0.085	4.12	0.012	1.274	1.025-1.582
LDL	0.184	0.082	3.21	0.026	1.243	1.002-1.538
Total cholesterol	0.152	0.068	3.79	0.017	1.204	1.010-1.436
Take aspirin regularly	-0.181	0.085	3.22	0.026	0.685	0.530-0.975
Sleeping	-0.344	0.117	6.85	0.006	0.578	0.514-0.887
Confidence	-0.415	0.178	4.48	0.010	0.522	0.427-0.918

**Table 2:** Multivariate logistic regression results of recurrence in patients with IS.

Factors	*B*	S.E.	Wald	*P*	OR	OR (95% CI)
Age	0.045	0.006	23.12	<0.001	1.036	1.018-1.055
Diastolic pressure	0.047	0.005	35.78	<0.001	1.040	1.022-1.055
Language disability	0.762	0.180	12.54	<0.001	2.169	1.460-2.221
Drinking	0.488	0.205	4.30	0.010	1.661	1.073-2.572
Triglycerides	0.216	0.085	4.12	0.012	1.274	1.025-1.582
Take aspirin regularly	-0.181	0.085	3.22	0.026	0.685	0.530-0.975
Sleeping	-0.344	0.117	6.85	0.006	0.578	0.514-0.887

**Table 3:** Area under ROC curve of the logistic regression model and related results.

AUC	95% CI	Accuracy	Sensitivity	Specificity	Youden's index
0.735	0.496-0.825	82.5%	63.2%	75.6%	38.2%

**Table 4:** Area under ROC curve of BP neural network and related results.

AUC	95% CI	Accuracy	Sensitivity	Specificity	Youden's index
0.796	0.658-0.912	86.8%	82.1%	80.5%	64.7%

## Data Availability

The datasets used during the current study are available from the corresponding author on reasonable request.
